# Artificial Intelligence Technology Driven Environmental Factors Extraction and Analysis Method in Traditional Clothing Handicraft

This article has been retracted.

**DOI:** 10.1155/2022/1883641

**Published:** 2022-10-12

**Authors:** Ran Tao, Qi Guo

**Affiliations:** ^1^Jilin Animation Institute, Changchun 130013, China; ^2^Academy of Fine Arts, Northeast Normal University, Changchun 130117, China

## Abstract

The application of artificial intelligence (AI) technology in the field of clothes can provide a good development mode and system under the social context of AI technology development. AI provides help for the development of intelligent clothing. Intelligent clothing is a high-tech product that integrates intelligent technology and clothing. It combines cutting-edge technologies in electronic information technology, sensor technology, textile science, and material science. In the extraction and analysis of environmental factors in clothing handicraft, AI technology has a considerable application prospect and a certain development potential. In order to improve the accuracy of environmental factors extraction in clothing handicraft, this paper uses convolutional neural network (CNN) to extract and analyze environmental factors in traditional clothing handicraft. We carried out experiments on the extraction of environmental factors in clothing handicrafts with pure color, few patterns, patterns, and complex background. The experimental results show that the CNN has a good effect on the extraction of environmental factors in clothing handicraft under different backgrounds. In addition, the model in this paper has good stability, accuracy, and feature extraction speed, which has high practical value and research significance.

## 1. Introduction

The fashion design trend of the 21st century will be based on the appearance of the fabric material as the conception basis, through the material to play out the distinctive characteristics, but also can convey the essence of the beauty of clothing. Decoration can not only sublimate the overall beauty of clothing but also highlight the important way of design concept and personality [1]. In the past decades, the emergence of the Internet has made a great contribution to the development of human society. Artificial intelligence (AI) has begun to appear in people's vision and integrated into all aspects of people's lives. It is known as the most groundbreaking technology in future science and technology. With the innovation of science and technology, the traditional clothing industry will inevitably be subjected to new changes and impacts. In the early years, some fashion designers applied high technology to fashion design, and the extraction of environmental factors in clothing also appeared in the public's view [2]. In the context of intelligent life, the combination of AI and clothing design will adapt to people's various clothing needs in the future, and gradually integrate into people's daily life to bring more convenience. Being a labor-intensive sector, the clothing business will have enormous profit potential once AI is implemented. By interpreting customer information, such as customer preferences and purchase histories, AI may use the well-known e-commerce and mobile commerce platforms to offer more appropriate products to online buyers, so as to create a truly personalized shopping experience [3, 4]. The combination of various technologies will inevitably lead to the use of new smart materials or wearable devices to improve the performance of products. When applying AI technology in smart clothing, it is necessary to consider not only the functionality of the clothing but also the comfort and safety of the human body when the fabric or wearable device touches the human skin, whether the clothing conforms to ergonomics, and whether the clothing is safe when wearing.

AI can also be involved in various jobs in the clothing industry, such as improving communication with customers by learning languages and helping companies talk to sellers. The garment sector can also benefit from AI technology's assistance in processing, analyzing, and predicting future consumption trends [5]. In the future, when AI is a necessity for China's economic growth, the garment sector can employ AI to complete industrial transformation and upgradation. The primary function of AI clothing as a functional article of clothing is to offer services to certain users [6]. Users will accept new products differently due to differences in their living conditions, social classes, and educational backgrounds. This necessitates that designers assess user cognition, product experience, and emotional acceptance of AI throughout the design process in order to satisfy users' psychological and physiological demands. Additionally, designers must keep up with the introduction of new technology, integrate it in real-time with scientific and technological advancements, and better cater to consumer needs [7].

The volume of clothes image data on the Internet has rapidly expanded as a result of the e-commerce for apparel's quick expansion. How to extract environmental factors from traditional clothing handicraft has become a research hotspot in recent years. There are now two different types of traditional ways for retrieving images of apparel. One is text-based image retrieval, which performs semantic matching on the text description of the clothing image [8, 9]. The other type is image retrieval based on image content, which extracts features from the color, texture, and other aspects of the image. However, these two methods have some limitations, and the artificial semantic labels for text description are very complicated [10]. However, the content features cannot fully reflect the rich visual features of the image, resulting in poor retrieval results [11]. At present, with the rapid development of deep learning technology and image processing technology, the powerful feature extraction ability of AI can be used to directly process images, which can eliminate the influence brought by different underlying features. According to statistics, the research interest has increased sharply since 2005, indicating that image extraction technology is gradually widely used in the field of clothing, and AI technology driven environmental factors extraction in traditional clothing handicraft has been further developed [12, 13].

Image segmentation and object extraction has been a hot topic in the field of computer vision and multimedia. Its application scope involves biomedicine, remote sensing aviation, industrial automation, and other fields. In recent years, the field of clothing gradually uses image extraction technology to extract clothing manual environmental features and process all kinds of clothing, and has made preliminary progress, which also shows that the use of AI technology to solve the problems in the clothing industry has attracted more and more attention and attention of AI research and clothing industry personnel [14]. From the perspective of garment contour and pattern extraction, many new garment styles are designed every year in the world, but few people have studied the extraction and analysis methods of environmental factors in traditional garment handicraft driven by AI technology. If the image extraction technology is used to extract the required clothing items from the clothing images, the second utilization of clothing styles can be realized. The clothing designers will be able to store the clothing styles electronically and extract their previous clothing design features easily. The construction of pattern database can also link the pattern database with the virtual platform to realize the independent personalized design of consumers [15, 16]. Traditional clothing is mainly made of ordinary fiber cutting and production, the main function is to cover the body, beautiful fashion. Intelligent clothing is mainly composed of intelligent materials, such as optical fiber and memory fiber. Intelligent clothing needs to consider the configuration of electronic components to ensure intelligence and wear comfort. For intelligent clothing combined with AI, the interactivity between clothing and AI, the availability of intelligent clothing materials, and supporting services should also be considered in the design.

It can be seen from the above that in order to improve the accuracy and efficiency of fashion image and contour extraction, many scholars use a combination of various algorithms [17]. In recent years, Fourier and clustering algorithms are widely used in fashion image style and contour extraction. Although the use of traditional algorithms cannot effectively complete the contour recognition of clothing background features, but to a large extent completed the extraction of clothing background features. Because of the diversity of clothing styles and background features, the existing single algorithm is usually suitable for the simple structure of clothing style map extraction. The stability and applicability of the algorithm still needs to be further improved for the extraction of garment background features with complex contour structure features [18]. Future smart clothing will be the product of the integration of various fields of technology and will have greater development potential.

In view of the mentioned problems, this paper uses convolutional neural network (CNN) to extract and analyze the environmental factors in traditional clothing handicrafts, and carries out experiments on the extraction of environmental factors in clothing handicrafts with pure color, few patterns, color, and complex background, respectively. The experimental results show that our model has better representation ability for high-level features formed by low-level feature learning, abstraction, and combination. We randomly take the average value of 1000 extraction times, and the result shows that feature extraction has a fast speed, which can meet the needs of daily image feature extraction. In view of the advantages of computing speed and storage space in feature extraction, CNN model ensures excellent feature extraction speed of the model, which has high theoretical value and research significance.

## 2. Related Works

The potential for traditional handicrafts to flourish sustainably was covered by Li et al. [19]. It is demonstrated through a review of the literature and an analysis of it that design science, as a link between the natural sciences and the humanities, seeks to advance key research techniques and instruments for the long-term sustainability of traditional handicrafts. This paper demonstrates that scientific design is the present and future of the sustainable development of traditional handicrafts, and presents five dynamic thinking methods and design strategies that provide the most direct method and theoretical foundation for the sustainable development of traditional handicrafts. According to Xue et al. [20], who investigated a unique fashion consumption theory of traditional handicraft mode based on the mature theories of planned behavior and self-concept theory, a new area for the study of slow fashion consumption has now been opened up. In order to improve product planning and marketing for traditional fashion businesses, the key drivers of the resurrection of the Chinese traditional handicraft industry are identified and elaborated.

Jiang [21] concentrated on the modeling approach of manufacturing resources relational database for the design and optimization of large-scale handicrafts in light of the issues that currently exist in the modeling of manufacturing resources. The manufacturing resource library is constructed as intended, and it is easy to retrieve many types of handicrafts. The experimental findings demonstrate an increase of 7.3% in the index efficiency of SQL AI for various sorts of handicrafts. By examining sample cases of Chinese traditional handicraft cultural brands, Xinchang and Jifeng [22] investigated how and why to develop traditional handicraft brands in the modern period. By establishing a distinctive brand identity, creating novel items, increasing new media exposure, and reviving Jiangsu region's handcraft tradition. This will help Jiangsu, and possibly the entire nation, preserve its traditional handicraft culture and advance it internationally. By examining the creative and aesthetic qualities of the handicraft, Osman et al. [23] established the identity of printed women's accessories. It is beneficial to emphasize the significance of national handicraft history because it is a significant component of human culture. A set of complementing fabrics for women's printing patterns is created by combining the design of the craft traditions of various nations with modern printing technology.

## 3. Models and Related Methods

### 3.1. Convolutional Neural Network

As science and technology have advanced quickly, AI has taken center stage. This technology is now widely used across a variety of industries and fills an essential role. The comprehensive application of AI technology in the clothing sector allows for a more rapid and accurate understanding of the fashion trend of garment attributes. Simultaneously, the use of AI to extract environmental factors from traditional clothing handicrafts can play a role in saving manpower and financial resources while achieving the objective of improving labor productivity. Traditional handicrafts and costumes advocate ecological spirit, symbolizing the harmonious coexistence between man and nature. Due to its unique attribute of handmade, it forms the characteristic branch of slow fashion, which marks the sustainable development trend in the field of fashion design.

The research of CNN originated from the visual cortex of the brain and was applied to the field of image recognition since 1980s [24, 25]. In the past decades, with the improvement of computer power and the increase of good datasets, CNN have achieved breakthrough levels in some complex computer vision tasks, often approaching or even sometimes exceeding human capabilities. In addition to visual tasks, CNN can also be applied to other tasks involving feature extraction stages, such as speech recognition and natural language processing. The main structure of CNN is composed of a large number of convolutional layers and pooling layers [26, 27]. The process of CNN processing the input image is shown in Figure 1. The convolutional layer simulates the local receptive fields of neurons in the visual cortex to translate and convolve the input image. Then the pooling layer reduces the dimension of the feature map obtained by the convolution layer to obtain a smaller feature map with more concentrated information. The operation is repeated for a certain number of times, and the final feature map is expanded into a one-dimensional tensor, which is input to the final classification layer for probabilistic output [28].

The most crucial part of CNN is the convolutional layer. Convolution is a mathematical operation that slides one function over another function and computes the integral of its dot product [29]. It is widely used in signal processing. The convolution layer is similar to the convolution in that it actually uses cross correlation. In the process of using the convolution layer to process the input image, the convolution kernel is actually used to extract local features by using the sliding average of the image.  Figure 2 shows the convolution process of the 2 × 2 convolution kernel for the input image matrix. The convolution kernel slides the input image from left to right and from top to bottom according to a predetermined step size and calculates the dot product sum of the convolution kernel and the corresponding window elements as the corresponding element value on the new feature map [30, 31]. The feature information extracted by the multilayer convolution process on the image corresponds to the basic texture features of the image to the abstract semantic features from top to bottom.

The pooling layer usually appears at the end of the feature map of a certain size and at the beginning of the downsampling layer [32]. The function of pooling layer is to reduce the size of feature map, reduce the amount of calculation and parameters, and prevent overfitting. Each neuron in the pooling layer is connected to the output of a limited number of neurons in the preceding layer that are situated in a constrained rectangular receptive field, just like the convolutional layer [33]. Different from the convolution layer, the neurons in the pooling layer do not contain weight parameters, and the neurons only process the mean or maximum value of the elements in the feature map. As shown in Figure 3, a 3 × 3 pooling kernel performs local mean processing on the feature map. Generally, the sliding step size of the pooling kernel is 2 from left to right and from top to bottom, so that the size of the feature map obtained after pooling is half of that before pooling [34, 35].

At the end of the network, the feature classification layer adopts a fully connected method for the feature information obtained after convolution and pooling [36]. As shown in Equation (1), where the output *x*_*i*_ of each category is mapped to [0, 1] after activation by softmax function to represent the probability of multiple classification, and the sum of probabilities of all categories is 1.

(1) $$\begin{array}{c} y\left(x_{i}\right)=\frac{\exp\left(x_{i}\right)}{\sum_{i=1}^{m}\exp\left(x_{i}\right)}. \end{array}$$

In order for the convolutional neural network to be able to approximate any function, the activation function is applied in the convolutional layer to improve its nonlinear representation capability. The Rectified Linear Unit (ReLu) shall be calculated to the reasonable satisfaction as shown in Equation (2), where *i* = 0.1, ⋯, *n* and *n* refers to the number of network layers. For the output *x*_*i*_ of layer *i*, the positive original value is output and the negative value is assigned zero [37]. Compared with other activation functions, there is no need to calculate exp(*x*_*i*_), and the output value is not centered at zero after activation. The ReLu function directly assigns zero to negative values, making this part of the neuron unable to be activated.

(2) $$\begin{array}{c} f\left(x_{i}\right)=\max\left(0,x_{i}\right) \end{array}$$

Leaky ReLu activation function improves the ReLu function to give a nonzero slope to all negative values to prevent this part of the neuron from failing to activate. The calculation formula is as follows:

(3) $$\begin{array}{c} y_{i}=\left\{\begin{array}{cc} x_{i} & \text{if }x_{i}\geq 0,\\ \frac{x_{i}}{a_{i}} & \text{if }x_{i}<0. \end{array}\right. \end{array}$$

In order to improve the accuracy of environmental factor feature extraction in traditional clothing handicraft, the clothing image data participating in the training were preprocessed with normalization and mean removal for subsequent numerical experiments. Normalization is also a way to simplify calculation. After transformation, the dimensionless expression is reduced to a dimensionless expression, so that indexes of different units or magnitude can be compared and weighted [38]. Normalization maps the data to the specified range reduces the difference of data values of each dimension, and reduces the influence on the classification experiment results caused by the large difference of data value range [39, 40]. Common normalization methods include feature standardization and simple scaling of image pixels. This paper adopts min-max normalization.

(4) $$\begin{array}{c} x_{\text{new}}=\frac{x-x_{\min}}{x_{\max}-x_{\min}}, \end{array}$$

where *x*_new_ is the new data value obtained after normalization, *x*_max_ is the maximum value of the sample data, and *x*_min_ is the minimum value of the sample data.

The mean removal operation means that the feature mean of all the images participating in training is subtracted from the feature mean of each image participating in training, so as to centralize the input data of each dimension to 0, so as to reduce the computational load. For *m* input samples, the *j*th pixel of sample *x*^(*i*)^ is represented as *x*_(*j*)_^(*i*)^, and the mean value of this pixel is calculated using the following formula:

(5) $$\begin{array}{c} \mu =\frac{1}{m}\overset{n}{\underset{i=1}{\sum }}x_{\left(j\right)}^{\left(i\right)}, \end{array}$$

where *μ* is the average vector of the whole training set data.

Color moment is a common algorithm to extract color features of images. It uses the concept of moments in linear algebra to represent the color distribution in images by moments. The formula of the color moment can be expressed as:

(6) $$\begin{array}{c} \mu_{i}=\frac{1}{N}\overset{N}{\underset{j=1}{\sum }}P_{i,j}, \end{array}$$

(7) $$\begin{array}{c} \sigma_{i}={\left(\frac{1}{N}\overset{N}{\underset{j=1}{\sum }}{\left(P_{i,j}-\mu_{1}\right)}^{2}\right)}^{1/2}, \end{array}$$

(8) $$\begin{array}{c} S_{i}={\left(\frac{1}{N}\overset{N}{\underset{j=1}{\sum }}{\left(P_{i,j}-\mu_{1}\right)}^{3}\right)}^{1/3}, \end{array}$$

where *P*_*i*,*j*_ represents the occurrence probability of pixels with gray level *j* in the *i*th color channel of the clothing image, and *N* represents the number of pixels in the image.

### 3.2. Combination of AI Technology and Extraction and Analysis of Environmental Factors in Traditional Clothing Handicraft

In the modern information age, intelligence has become a trend of the current era. The creation and use of new scientific and technological materials offers a significant assurance for the continued growth of the apparel sector. Additionally, clothing will play a significant role in the clothing industry. The development of AI has also opened up endless possibilities for clothing. From the perspective of the development prospect of AI in fashion design, the transformation of the fashion industry is inevitable, as is the combination with science and technology. The marriage of AI and apparel can keep up with the development of the quick-paced age, offer people more comfortable and convenient life services, and has a promising future for market growth. The clothing industry is bound to help the development of AI industry usher in its own era in the future [41]. The traditional clothing industry has also ushered in the wave of reform and upgrading. The emergence of AI technology can effectively solve the pain points of the clothing industry, especially in the field of promoting the clothing industry to achieve flexible production, AI technology will help more enterprises to transform efficiently.

The use of computer technology and human-computer interaction technology can effectively improve the efficiency of manufacturing; enhance the flexibility of all aspects of work. Therefore, AI technology has the potential to accelerate economic growth, enhance the environment for the growth of the clothing business, and change the way the clothing industry has traditionally developed. The garment industry is labor intensive, and the adoption of AI technology can expand the profit margin, especially in the sales of the garment industry. To a certain extent, this cannot only break the development mode and mechanism of the traditional clothing industry but also effectively reform the sales and management work of the traditional clothing industry, and fundamentally promote the improvement of work quality in all aspects. It can be seen that the extraction and analysis methods of environmental factors in traditional clothing handicraft under AI technology have a considerable prospect, which should be paid enough attention to and effective measures should be taken to complete their own tasks.

People have progressed from the level of material pursuit to the level of quality of life in the actual course of life, from the standpoint of the market and future development prospects, and the collocation of clothing and surrounding environment can meet people's needs for quality of life to a certain extent. In the rapid development of our economy and science and technology, the development of environmental factors extraction in costume handicraft has become an inevitable trend. The application of AI technology in the extraction of environmental factors in traditional clothing handicraft can form a good development prospect. The effect of clothing design and manufacture can be successfully optimized by the use of AI technology in the extraction of environmental parameters in traditional clothing handcraft. The convenience of design, the functionality of intelligent clothing, the user's operation process and operation links, and the provision of user support services can all be effectively improved with the aid of AI technology, particularly in the field of design. It is feasible to adopt AI technology in the extraction of environmental factors in traditional clothing handicraft, which should be actively promoted and applied.

We first input the image to be processed into the network model for forward propagation, and then retrieve image characteristics through sampling, in order to fully extract garment environmental elements. To achieve the extraction of environmental factors in traditional clothing handicraft, the results of the softmax classifier based on the CNN model are hashed and then passed into the relevant index database for an approximatively nearest neighbor search. The image results are then returned sorted by similarity. The overall structure of the model in this paper is shown in Figure 4. In the process of clothing feature extraction, the input image is subjected to the same feature extraction and mapping, and the index library of the samples with high similarity to the input image is obtained by comparison. The binary hash code of the input image and the hash code in the library are used to measure the similarity one by one, so as to achieve the fast feature extraction of the clothing image.

## 4. Numerical Experiments

In this paper, Java language is used to implement an AI technology-driven extraction and analysis method for environmental factors in traditional clothing handicraft. The detailed test environment is shown in Table 1. Images of the garments used in the tests were downloaded from websites such as Taobao and Baidu.

The evaluation index of feature extraction of environmental factors is generally the average precision MAP calculation. True positive (TP), false positive (FP), and false negative (FN) should be used to calculate the evaluation index, and the calculation formula is as follows:

(9) $$\begin{array}{c} \text{TP}=\underset{{\text{Iou}}_{i}>{\text{Iou}}_{\text{threshold}}}{\sum }1, \end{array}$$

(10) $$\begin{array}{c} \text{FP}=\underset{0<{\text{Iou}}_{i}\leq {\text{Iou}}_{\text{threshold}}}{\sum }1, \end{array}$$

(11) $$\begin{array}{c} \text{FN}=\underset{{\text{Iou}}_{i}=0}{\sum }1, \end{array}$$

where Iou_threshould_ is the preassumed threshold of intersection and union ratio, Iou_*i*_ is the intersection and union ratio of the *i*th detection box, and *n* is the total number of detection boxes. Precision and recall can be calculated as follows:

(12) $$\begin{array}{c} \text{Precision}=\frac{\text{TP}}{\text{TP}+\text{FP}}, \end{array}$$

(13) $$\begin{array}{c} \text{Recall}=\frac{\text{TP}}{\text{TP}+\text{FN}}, \end{array}$$

By testing 20,000 random samples of clothing image set, the extraction accuracy of softmax classifier is 92.71%. Experiments show that CNN network has a good pertinence for the extraction of environmental factors in traditional clothing handicraft, and can achieve the expected extraction effect.  Figure 5 shows the extraction effect of environmental factors in solid-color clothing handicraft. It can be found that even if the color of clothes is similar to the environment, the surrounding environment of clothes can also be extracted.

We further confirmed the impact of various datasets on the precision of feature extraction. The detection accuracy produced by experiment is displayed in Table 2 for the verification data.

The experimental findings demonstrate that as the dataset is expanded, feature extraction accuracy increases and gradually tends to stabilize; ensuring that the model will also have a certain degree of stability for the dataset of images of oversized clothing. Figures 6 and 7, respectively, show the extraction effect of environmental factors in the traditional costume handicraft with a small number of patterns and the extraction effect of environmental factors in the traditional costume handicraft with color. The numerical results show clearly that our model has better representation ability for high-level features formed by low-level feature learning, abstraction and combination.

We randomly take the average value of 1000 times of extraction time, and the average time of feature extraction is 3.2416 s. Feature extraction has a fast speed and can meet the needs of daily image feature extraction. In view of the advantages of computing speed and storage space of CNN model in feature extraction, the excellent feature extraction speed of the model is guaranteed.  Figure 8 shows the extraction effect of environmental factors in clothing handicraft under complex background. The experimental results show that the CNN model cannot only ensure the extraction speed but also efficiently extract clothing background features under complex background.

As a functional clothing, the main purpose of AI clothing is to provide services for specific users, and can serve different needs, and can withstand the subjective choice of the buyer's market. Due to the different living environment, social class and educational background of users, their acceptance of new products will also be different. Designers are required to evaluate user cognition, product experience, and emotional acceptance of AI in the process of design, so as to meet the psychological and physical needs of customers. At the same time, designers also need to pay attention to the release of new technology, real-time integration with the development of science and technology, better adapt to the needs of users.

## 5. Conclusions

In the overall design effect of clothing beauty, clothing handicraft is often an important means to beautify clothing. Based on the revolution wave of AI, the future garment industry will face both opportunities and challenges. Most designers generally hold the clothing modeling characteristics, material properties, and the use of color. In fact, in the field of fashion design, a variety of artistic and technical means should be used to make clothing more perfect and more distinctive. In this study, trials are conducted to determine how environmental elements can be extracted from clothing handicrafts with simple color schemes, few patterns, and complex backgrounds. The experimental results show that the convolutional neural network has a good effect on the extraction of environmental elements in apparel handicraft under varied backgrounds. In addition, the model has good stability, accuracy, and retrieval speed, which has high practical value and research significance.

Future work can also extract features from clothing with more colors and textures. On the basis of the development of the fashion pattern database, the extracted fashion pattern data information can also be fitted to the virtual image, so that the user can experience a more real 3D fitting effect. In addition to the optimization of the virtual fitting process of professional equipment, the high definition image brought by the upgrading of the clothing feature extraction technology. In the future, modern fashion database can be connected with traditional clothing database, and virtual design experiment adjustment can be carried out through virtual platform, intelligent design, and other systems to complete more excellent design works.

## Figures and Tables

**Figure 1:** Image processing process of convolutional neural network.

**Figure 2:** Convolution process of convolution kernel.

**Figure 3:** Schematic diagram of the pooling process.

**Figure 4:** Overall framework of environmental factors extraction in traditional clothing handicraft based on GNN.

**Figure 5:** Environmental factors in the pure color clothing handicraft extraction effect.

**Figure 6:** Extraction effect of environmental factors in traditional clothing handicraft with few patterns.

**Figure 7:** Extraction effect of environmental factors in traditional color and dress handicraft.

**Figure 8:** Extraction effect of environmental factors in clothing handicraft under complex background.

**Table 1:** Extraction and analysis of environmental factors in traditional clothing handicraft test environment.

Hardware environment	CPU: Intel core i3-2330M, memory: 4 GB
Software environment	Windows 10, Tomcat 7.0, and MySQL 5.5
Development environment	JDK1. 7, OpenCV 2.4, and MyEclipse 10.0
System framework	Struts2.0, spring, and MyBatis

**Table 2:** Data volume and feature extraction accuracy.

Amount of experimental data	Feature extraction accuracy
50000	0.8842
100000	0.9056
150000	0.9213
20000	0.9286
250000	0.9349
300000	0.9398

## Data Availability

The data used to support the findings of this study are available from the corresponding author upon request.

## References

[1] Li Z., Rau P. L. P., Huang D. (2020). Who should provide clothing recommendation services: Artificial Intelligence or Human Experts?. *Journal of Information Technology Research (JITR)*.

[2] Wei X. The application and development of artificial intelligence in smart clothing.

[3] Ahsan M., Hon S. T., Albarbar A. (2020). Development of novel big data analytics framework for smart clothing. *IEEE Access*.

[4] Li Q., Xue Z., Wu Y., Zeng X. (2022). The status quo and prospect of sustainable development of smart clothing. *Sustainability*.

[5] Liu Y., Chen Y., Ding W., Yang X., Qu C. (2022). The research and application of artificial intelligence in smart clothing with Internet of Things in healthcare. *Innovative Computing*.

[6] Kim H. S., Lee J. H., Lee H. D. (2021). Development of personalized clothing recommendation service based on artificial intelligence. *Smart Media Journal*.

[7] Yan L., Liu W. Garment textile correction system based on artificial intelligence under computer parameter optimization design.

[8] Papachristou E., Chrysopoulos A., Bilalis N. (2021). Machine learning for clothing manufacture as a mean to respond quicker and better to the demands of clothing brands: a Greek case study. *The International Journal of Advanced Manufacturing Technology*.

[9] Jian S. (2022). Virtual reality technology facilitates customized clothing design in C2M business model. *Smart Communications, Intelligent Algorithms and Interactive Methods*.

[10] Zhang X., Deng Z. (2021). An improved method of clothing image classification based on CNN. *International Journal of Advanced Networking and Applications*.

[11] Wang F. Application of artificial intelligence-based video image processing technology in security industry.

[12] Zhong J., He B. Application of big data analysis and image processing technology in athletes training based on intelligent machine vision technology.

[13] He Y., Hu C., Li H. (2022). A flexible image processing technique for measuring bubble parameters based on a neural network. *Chemical Engineering Journal*.

[14] Patel K., Parmar B. (2022). Assistive device using computer vision and image processing for visually impaired; review and current status. *Disability and Rehabilitation: Assistive Technology*.

[15] Li H., Xu L., Shi Z., Wang X., Li J., Manogaran G. Research on environmental assessment method of meteorological observation station detection based on panoramic image processing.

[16] Muhammad N. A., Fatima R. (2022). Role of image processing in digital forensics and cybercrime detection. *International Journal of Computational and Innovative Sciences*.

[17] Zhang L., Zhang L., Zhang L. (2018). Application research of digital media image processing technology based on wavelet transform. *EURASIP Journal on Image and Video Processing*.

[18] Zhang X., Dahu W. (2019). Application of artificial intelligence algorithms in image processing. *Journal of Visual Communication and Image Representation*.

[19] Li W. T., Ho M. C., Yang C. (2019). A design thinking-based study of the prospect of the sustainable development of traditional handicrafts. *Sustainability*.

[20] Xue X., Caiguo X., Yi L., Chenxia M. (2022). Consumption of traditional handicraft fashion: motivations, intentions and behaviours of Chinese consumers. *Cleaner and Responsible Consumption*.

[21] Jiang Y. Design and optimization of large-scale traditional handicraft database based on SQL model.

[22] Xinchang O., Jifeng X. Digitalization and visual platform build-up of traditional handicraft culture in Jiangsu, Province.

[23] Osman S. M., Khalil D. A. H., Ibrahim N. M. (2022). The national handicraft heritage as a source for establishing a printed fabrics identity for use in women clothing accessories. *International Design Journal*.

[24] Kattenborn T., Leitloff J., Schiefer F., Hinz S. (2021). Review on convolutional neural networks (CNN) in vegetation remote sensing. *ISPRS Journal of Photogrammetry and Remote Sensing*.

[25] Liu Y., Pu H., Sun D. W. (2021). Efficient extraction of deep image features using convolutional neural network (CNN) for applications in detecting and analysing complex food matrices. *Trends in Food Science & Technology*.

[26] Alhichri H., Alswayed A. S., Bazi Y., Ammour N., Alajlan N. A. (2021). Classification of remote sensing images using EfficientNet-B3 CNN model with attention. *IEEE Access*.

[27] Dong P., Zhang H., Li G. Y., Gaspar I. S., NaderiAlizadeh N. (2019). Deep CNN-based channel estimation for mmWave massive MIMO systems. *IEEE Journal of Selected Topics in Signal Processing*.

[28] Khan A., Sohail A., Zahoora U., Qureshi A. S. (2020). A survey of the recent architectures of deep convolutional neural networks. *Artificial Intelligence Review*.

[29] Tulbure A. A., Tulbure A. A., Dulf E. H. (2022). A review on modern defect detection models using DCNNs - deep convolutional neural networks. *Journal of Advanced Research*.

[30] Arshad H., Khan M. A., Sharif M. I. (2022). A multilevel paradigm for deep convolutional neural network features selection with an application to human gait recognition. *Expert Systems*.

[31] Ali A., Zhu Y., Zakarya M. (2022). Exploiting dynamic spatio-temporal graph convolutional neural networks for citywide traffic flows prediction. *Neural Networks*.

[32] Dong Y., Liu Q., Du B., Zhang L. (2022). Weighted feature fusion of convolutional neural network and graph attention network for hyperspectral image classification. *IEEE Transactions on Image Processing*.

[33] Wisniewski M., Rana Z. A., Petrunin I. (2022). Drone model classification using convolutional neural network trained on synthetic data. *Journal of Imaging*.

[34] Yang B., Zhang Z., Yang C. Q. (2022). Identification of species by combining molecular and morphological data using convolutional neural networks. *Systematic Biology*.

[35] Umer M., Ashraf I., Ullah S., Mehmood A., Choi G. S. (2022). COVINet: a convolutional neural network approach for predicting COVID-19 from chest X-ray images. *Journal of Ambient Intelligence and Humanized Computing*.

[36] Rahimilarki R., Gao Z., Jin N., Zhang A. (2022). Convolutional neural network fault classification based on time-series analysis for benchmark wind turbine machine. *Renewable Energy*.

[37] Herrmann J., Llima S. M., Remm A. (2022). Realizing quantum convolutional neural networks on a superconducting quantum processor to recognize quantum phases. *Nature Communications*.

[38] Castillo-Barnes D., Jimenez-Mesa C., Martinez-Murcia F. J., Salas-Gonzalez D., Ramírez J., Górriz J. M. (2022). Quantifying differences between affine and nonlinear spatial normalization of FP-CIT SPECT images. *International Journal of Neural Systems*.

[39] Lin Y., Wang H., Wang S. (2022). Roles of silicon content and normalization temperature on cold workability and recrystallization of high-grade non-oriented silicon steel. *Crystals*.

[40] Talat N., Alsadoon A., Prasad P. W., Dawoud A., Rashid T. A., Haddad S. (2022). A novel enhanced normalization technique for a mandible bones segmentation using deep learning: batch normalization with the dropout. *Multimedia Tools and Applications*.

[41] Majumdar A., Garg H., Jain R. (2021). Managing the barriers of industry 4.0 adoption and implementation in textile and clothing industry: interpretive structural model and triple helix framework. *Computers in Industry*.

